# Deep Learning-Based Computed Tomography Features in Evaluating Early Screening and Risk Factors for Chronic Obstructive Pulmonary Disease

**DOI:** 10.1155/2022/5951418

**Published:** 2022-08-18

**Authors:** Changhong Zhang, Jianhua Liu, Liang Cao, Gaixia Feng, Zhihua Zhang, Mengmeng Ji, Yaping Zhang

**Affiliations:** ^1^Department of Respiratory and Critical Care Medicine, The First Affiliated Hospital of Hebei North University, Zhangjiakou 075000, Hebei, China; ^2^Department of Medical Imaging, The First Affiliated Hospital of Hebei North University, Zhangjiakou 075000, Hebei, China

## Abstract

This research aimed to investigate the diagnostic effect of computed tomography (CT) images based on a deep learning double residual convolution neural network (DRCNN) model on chronic obstructive pulmonary disease (COPD) and the related risk factors for COPD. The questionnaire survey was conducted among 980 permanent residents aged ≥ 40 years old. Among them, 84 patients who were diagnosed with COPD and volunteered to participate in the experiment and 25 healthy people were selected as the research subjects, and all of them underwent CT imaging scans. At the same time, an image noise reduction model based on the DRCNN was proposed to process CT images. The results showed that 84 of 980 subjects were diagnosed with COPD, and the overall prevalence of COPD in this epidemiological survey was 8.57%. Multivariate logistic regression model analysis showed that the regression coefficients of COPD with age, family history of COPD, and smoking were 0.557, 0.513, and 0.717, respectively (*P* < 0.05). The diagnostic sensitivity, specificity, and accuracy of DRCNN-based CT for COPD were greatly superior to those of single CT and the difference was considerable (*P* < 0.05). In summary, advanced age, family history of COPD, and smoking were independent risk factors for COPD. CT based on the DRCNN model can improve the diagnostic accuracy of simple CT images for COPD and has good performance in the early screening of COPD.

## 1. Introduction

Chronic obstructive pulmonary disease (COPD) is a common, preventable, and treatable chronic airway inflammatory disease characterized by persistent respiratory symptoms and airflow restriction [1]. Patients usually present with long-term, repeated, and gradually aggravating cough and sputum and even involve the heart in serious cases, presenting symptoms such as palpitation, limb edema, and chest tightness [2–4]. COPD generally develops from chronic bronchitis and emphysema and further develops into pulmonary heart disease, respiratory failure, pulmonary encephalopathy, and systemic complications [5]. In recent years, COPD has become one of the three major death factors worldwide and the fatality rate is second only to coronary heart disease and cerebrovascular disease. Clinical observation shows that COPD is most common among smokers, followed by family history, air pollution, and irritating gas [6, 7]. Generally, the pulmonary function can be detected and diagnosed early in the vast majority of patients. If cough, sputum, and wheezing occur frequently, especially for long-term smokers and those exposed to risk factors, vigilance must be raised [8].

At present, lung function examination of patients is the gold standard for the diagnosis of COPD, which can detect early small airway lesions, determine whether the airflow restriction is completely reversible and severe, determine whether there are signs of emphysema, and understand lung residual volume, alveolar diffusion function, and alveolar membrane permeability [9, 10]. X-Ray examination can display the texture features of both lungs, rib spacing, and lung permeability and is easy to operate and cheap, but the diagnostic effect is general, and there are misdiagnoses and missed diagnoses [11]. Echocardiography can be used to judge the pulmonary artery pressure, understand whether the pulmonary artery widens or increases resistance, and monitor changes in pressure and resistance of the right ventricle and right atrium, with the advantages of no radiation and simple operation [12]. Chest CT examination is an auxiliary method commonly used in COPD screening at present. It can reflect changes in the overall lung function of patients from the lung structure and function at the same time, with high diagnostic sensitivity. Nevertheless, it has certain limitations and is only suitable for patients with serious diseases [13].

Imaging technology is the most widely used diagnostic method in the clinic. However, due to a variety of objective factors, the images often have noise, artifacts, and other problems, resulting in a poor image quality, which cannot help doctors carry out a more accurate evaluation. Therefore, in many cases, the mathematical model is needed to enhance the image first to improve the image quality [14]. Deep learning refers to a collection of algorithms that use various machine learning algorithms to solve various problems, such as images and texts, on multilayer neural networks. It is classified into neural networks, whose core is feature learning and obtaining hierarchical feature information through hierarchical networks, to solve important problems requiring manual design of features in the past, and it is widely used in the field of medical images [15]. Higaki et al. [16] developed a deep learning reconstruction (DLR) method to reduce image noise by integrating the deep convolutional neural network (DCNN) into CT image reconstruction. It was ultimately found that on DLR images that the image noise is lower and the high contrast spatial resolution and task-based detectability are better than those reconstructed using other state-of-the-art techniques. Sun et al. [17] proposed a single degradation-aware deep learning framework to predict sharp CT images by understanding the difference in degradation in the frequency and image domains. Peak signal-to-noise ratio, structural similarity, and visual results demonstrate that this method outperforms classical deep learning-based reconstruction methods in terms of effectiveness and scalability.

In summary, early screening for COPD is still a topic that needs to be explored. Based on this, in this research, a questionnaire survey was conducted among 980 permanent residents aged ≥40 who underwent a physical examination. Among them, 84 patients who were diagnosed with COPD and volunteered to participate in the experiment and 25 healthy people were selected as the research subjects, and all of them underwent CT imaging scans. At the same time, an image noise reduction model based on the DRCNN was proposed to process CT images to deeply explore the early screening effect and related risk factors of COPD combined with deep learning and CT images.

## 2. Materials and Methods

### 2.1. Epidemiological Survey Samples

A total of 980 permanent residents aged ≥40 years who underwent a physical examination at a hospital from January 2021 to December 2021 were selected as subjects. Inclusion criteria were as follows: those aged above 39; those with complete basic information; and those who were able to read and write Chinese and communicate without barriers. Exclusion criteria were as follows: those with mental or neurological disorders; those with impaired auditory, visual, and verbal expression and poor communication; and those who did not want to participate. This research was approved by the ethics committee of the hospital. All the subjects were informed and gave their consent to participate in the study.

Among 980 subjects, 84 patients with confirmed COPD and 25 healthy volunteers were selected as study samples. The inclusion criteria were as follows: those aged over 40 years old; those with a history of exposure to risk factors; and those with complete clinical data. The exclusion criteria were as follows: those who had combined pleural effusion; cognitive impairment; complications with other chronic respiratory diseases; and poor inspection compliance.

### 2.2. Clinical Data Collection

Data collection investigators will be uniformly trained and qualified. According to the *Overview of The Surveillance Content and Methods of Chronic Obstructive Pulmonary Disease in Chinese Residents*, a self-made questionnaire survey was conducted among eligible elderly people before the physical examination, including gender, smoking, age, education level, marital status, BMI, family history of COPD, and heating method.

### 2.3. Pulmonary Function Test

For pulmonary function examination, all subjects sat, stood upright, and breathed smoothly before the examination. Lung volume and ventilatory function were measured by a German Jaeger pulmonary function detector. Forced vital capacity and forced expiratory volume were tested for one second. The examination procedures and interpretation were performed by technicians and physicians with more than two years of pulmonary function examination experience.

The diagnosis of COPD was based on the relevant criteria in the *Guidelines for Diagnosis and Treatment of Chronic Obstructive Pulmonary Disease* (*2013 Revision)*: FEV1/FVC < 70% after inhaling bronchodilators. According to the relevant content in the 9th edition of *Internal Medicine*, the severity of airflow restriction was graded by GOLD grading and FEV1 descent. The percentage of FEV1 in lung function ≥80% was grade 1 (mild), 50%–79% was grade 2 (moderate), 30%–49% was grade 3 (severe), and <30% was grade 4 (very severe).

### 2.4. CT Examination Methods

Lung CT examinations were performed on 84 COPD patients and 25 normal volunteers with dual-source CT apparatus. Prior to the examination, the patient was instructed to take deep a breath and hold their breath at the end of the examination. During the examination, the patient was in a supine position and scanned from the tip of the lung to the bottom of the lung at the end of the deep inspirations. The parameters were set as follows: the voltage was 120 kV, the current was 140 mA, the collimator was set at 64 × 0.5 mm, the pitch was 0.5, layer thickness was 0.5 mm, layer spacing was 0.5 mm, and the matrix was 512 × 512. The obtained images were transmitted to workstations for processing and independently diagnosed by two senior physicians.

### 2.5. Image Denoising Model Based on Deep Learning

The DRCNN model [18] is mainly composed of a projection domain element, intermediate domain element, and image domain element. The projection domain unit is used to denoise the projected data, the middle domain unit is used to decode the denoised image into the CT image to be processed, and the image domain unit is used to further improve the image quality (Figure 1).

If the original projection data are *p* and the normal dose projection data are *q*, then the function *H* that maps *p* to *q* can be expressed as follows:

(1) $$\begin{array}{c} H:p⟶q. \end{array}$$

In the past, a fully connected layer was used to carry out mapping operations, but such calculations were too large. Therefore, a filtering back projection module was introduced to replace the fully connected layer.

(2) $$\begin{array}{c} K:H\left(p\right)⟶K\left(H\left(p\right)\right). \end{array}$$

In formula (2), *K*(*H*(*p*)) denotes that the filtering back projection module transforms the denoised CT image *H*(*p*) to obtain a better CT image. To better improve the image quality, the mapping function *H*^*∗*^ of the image domain unit is set as follows:

(3) $$\begin{array}{c} H{}^{*}:K\left(H\left(p\right)\right)⟶K\left(q\right). \end{array}$$

In formula (3), *K*(*q*) is the normal reference image. Then, mean square error (MSE) is introduced as the objective optimization function of the DRCNN model.

(4) $$\begin{array}{c} Z_{DR}=\alpha_{1}Z_{1}\left(H\left(p\right),q\right)+\alpha_{2}Z_{2}\left\{H^{*}\left(K\left(H\left(p\right),q\right)\right)\right\}. \end{array}$$

In formula (4), *K*(*H*(*p*)) represents the image obtained by image domain processing, *Z*_1_ represents the MSE loss of the projection domain subnet minimized, *Z*_2_ represents the MSE loss of the image domain subnet minimized, *α*_1_ represents the balance coefficient of the projection domain subnet, and *α*_2_ represents the balance coefficient of the image domain subnet. Then, the total variation (TV) is introduced into the objective optimization function, so the TV loss of the final output image can be expressed as follows:

(5) $$\begin{array}{c} K{\left(H\left(p\right)\right.}_{TV}=\sum_{i}\Lambda_{i}K\left(H\left(p\right)\right.. \end{array}$$

In formula (5), Λ_*i*_ represents the discrete gradient operator. Given training data {*p*_*i*_, *q*_*i*_}_*i*∈Π_, the DRCNN optimization model can be expressed as follows:

(6) $$\begin{array}{c} \left\{H_{1}^{\propto },H_{2}^{\propto }\right\}=\underset{H_{1},H_{2}}{\text{argmin}}\left\{\alpha_{1}Z_{1}\left(H\left(p\right),q\right)+\alpha_{2}Z_{2}\left\{H^{*}\left(K\left(H\left(p\right),q\right)\right)\right\}+\alpha_{3}Z_{TV}\left(K\left(H\left(p\right)\right.\right.\right\}. \end{array}$$

In formula (6), *α*_3_ is the weighting coefficient of TV loss.

### 2.6. Image Quality Evaluation Indexes

The convolutional neural network model (CNN) [19] and residual network model (ResNet) [20] were introduced for comparison with the improved DRCNN model that is proposed in this research.

Normalized mean absolute distance (NMAD), root mean square error (RMSE), and peak signal-to-noise ratio (PSNR) were calculated to evaluate the image quality.

It is assumed that the reconstructed image is *l*_1_, the true image is *l*_0_, and the total number of image pixels is *M*; then,

(7) $$\begin{array}{c} \text{NMAD}=\frac{\sum_{i=1}^{M}\left|l_{0}\left(i\right)-l_{1}\left(i\right)\right|}{\sum_{i=1}^{M}\left|l_{0}\left(i\right)\right|},\\ \text{RMSE}=\sqrt{\frac{\sum_{i=1}^{M}{\left|l_{0}\left(i\right)-l_{1}\left(i\right)\right|}^{2}}{M}},\\ \text{PSNR}=10{\text{log}}_{10}\left[\frac{{\text{Max}}^{2}\left(l_{0}\right)}{\sum_{i=1}^{M}{\left|l_{0}\left(i\right)-l_{1}\left(i\right)\right|}^{2}|M}\right]. \end{array}$$

### 2.7. Statistical Methods

Statistical analysis data were analyzed by SPSS 23.0 statistical software package, count data were described by frequency or proportion, and comparisons between groups were performed by *χ*^2^ test. The influencing factors of COPD were analyzed by a multivariate logistic regression model. All tests were two-sided with *a* = 0.05.

## 3. Results

### 3.1. Survey Sample General Information

In Figure 2, in terms of gender, the number of female (553) was greatly superior to that of male (427). The number of smokers (518) was slightly higher than that of nonsmokers (462). In terms of age, the number of cases from 56 to 69 years old was the largest (433), followed by > 69 years old (289) and 40–55 years old (258). In terms of education level, the number of students with a qualification of high school or below was the highest (622), followed by college degree (253) and bachelor's degree or above (105). In terms of marital status, the number of married people was the highest (883), while the numbers of divorced people (21), single people (24), and widowed people (52) were the lowest. For BMI, those with 18.5–23.9 kg/m^2^ cases (471) were the highest, followed by those with >23.9 kg/m^2^ (329) and <18.5 kg/m^2^ (180 patients). In terms of family history of COPD, 137 patients had a family history and 843 had no family history. Coal (406) and natural gas (311) were the most popular methods of heating, followed by firewood (145).

### 3.2. Comparison of Prevalence Rates under Different Sociological Data

In 980 participants, 84 were diagnosed with COPD, so the overall prevalence was 8.57%. Further comparison of prevalence differences under different sociological data in Figure 3 shows that among 84 patients with the disease, 49 were male and 35 were female, and the prevalence rate of male (11.48%) was greatly superior to that of female (6.33%) (*P* < 0.05). The prevalence in smokers (11.58%) was greatly superior to that in nonsmokers (5.19%) (*P* < 0.05). There were 11 patients aged 40–55, 27 patients aged 56–69, and 36 patients aged >69 years old. The prevalence rate in those > 69 years old (12.46%) was greatly superior to that in those 40–55 years old (4.26%) and 56–69 years old (6.24%) (*P* < 0.05). In terms of educational level, 53 patients had a high school degree or below, 23 had a junior college degree, and 8 had a bachelor's degree or above. There was no notable difference in the prevalence rate of high school degree or below (8.52%), junior college degree (9.09%), or bachelor's degree (7.62%) (*P* > 0.05). There were 79 married patients, 0 divorced patients, 0 unmarried patients, and 5 widowed patients. There was no notable difference between the prevalence in married patients (8.95%) and widowed patients (9.62%) (*P* > 0.05). There were 20 patients with BMI < 18.5 kg/m^2^, 12 with BMI of 18.5–23.9 kg/m^2^, and 62 patients with BMI > 23.9 kg/m^2^. The prevalence of BMI > 23.9 kg/m^2^ (18.84%) was greatly superior to that of BMI < 18.5 kg/m^2^ (11.11%) and BMI 18.5–23.9 kg/m^2^ (6.67%), and the difference was considerable (*P* < 0.05). There were 61 cases with family history and 23 cases with no family history. The prevalence of family history (44.53%) was greatly superior to that of no family history (2.73%). There were 42 cases using coal, 29 cases using natural gas, 13 cases using firewood, and the rest were free of illness. There was no notable difference in the prevalence of coal (10.34%), natural gas (9.32%), and firewood (8.97%) (*P* > 0.05).

### 3.3. Multivariate Logistic Regression Analysis of COPD Occurrence

According to *χ*^2^ test results, normalization was carried out. Gender (male = 1, female = 0), age (> 69 years old = 2, 56–69 years old = 1, 40–55 years old = 0), BMI (< 18.5 kg/m^2^ = 0, 18.5–23.9 kg/m^2^ = 1, >23.9 kg/m^2^ = 2), family history of COPD (yes = 1, no = 0), and smoking (urban = 1, rural = 0) were taken as independent variables, and multivariate logistic regression analysis was performed with COPD as the dependent variable.  Table 1 shows that there was no significant correlation between COPD and sex or BMI. The regression coefficients of age, family history of COPD, and smoking were 0.557, 0.513, and 0.717, respectively (*P* < 0.05).

### 3.4. Comparison of Performance Indexes of Different Algorithms

In Figure 4, the NMAD and PSNR of the DRCNN model were greatly superior to those of the CNN model and ResNet model, and the differences were considerable (*P* < 0.05). The MSE of the DRCNN model was significantly smaller than that of the CNN model and ResNet model, and the difference was considerable (*P* < 0.05).

Figure 5 shows the CT image processing results of different algorithms. The quality of the original image was poor, the tissue display was not clear, and there were artifacts and noise. The clarity of images processed by the CNN model was significantly improved, but the details cannot be reflected due to the exposure transition. The image processed by the ResNet model had some changes in color balance, and there were still some artifacts and noises. After DRCNN model processing, the image artifact and noise were greatly reduced, and the sharpness was significantly improved. Meanwhile, there was no overexposure problem in DRCNN model processing, and the overall quality was the best.

### 3.5. CT Imaging Findings of COPD

Figure 6 shows the CT image data of a patient with COPD (male, 75 years old). CT showed two lung texture increases and thickening, partial lung transmittance increased, irregular patchy density increased in the posterior basal segment of the left lower lung, and some edges were clear. Coronary calcification was visualized. There were two slight pleural thickenings.

### 3.6. Comparison of Diagnostic Results between CT and Single CT Based on the DRCNN Model

With known results as the gold standard, the diagnostic sensitivity, specificity, and accuracy of DRCN-based CT and single CT for COPD were calculated, and the results are shown in Figure 7. The diagnostic sensitivity, specificity, and accuracy of DRCNN-based CT for COPD were greatly superior to those of single CT, and the difference was considerable (*P* < 0.05).

## 4. Discussion

COPD is a respiratory disease with a high incidence. The early symptoms are not obvious, and it is difficult to attract the attention of patients. When diagnosed, most patients progress to the middle and late stages, and the cure rate is greatly reduced. The clinical mechanism related to the occurrence of COPD is still unclear and may be related to a variety of factors, such as smoking, sex, heating method, and family history [21]. In order to further clarify the epidemiological characteristics of COPD, 980 permanent residents aged ≥ 40 who underwent physical examination were selected as the research subjects for a questionnaire survey. First, 84 of the 980 survey samples were finally diagnosed with COPD, so the total prevalence of this epidemiological survey was 8.57%, which was similar to the statistical data of Fang et al. [22] on the prevalence of COPD among people over 40 years old in 7 provinces and cities in China (3.9%–13.7%). Thus, the prevalence of COPD in this region was in the middle.

Prevalence was then analyzed. The prevalence rate of male (11.48%) was greatly superior to that of female (6.33) (*P* < 0.05), which is similar to the results of Occhipinti et al. [23]. The analysis may be related to the high number of male smokers. The prevalence in smokers (11.58%) was greatly superior to that in nonsmokers (5.19%) (*P* < 0.05), which is consistent with previous literature studies [24]. Among the 84 patients, 11 were aged 40–55 years, 27 were aged 56–69 years, and 36 were older than 69 years. The prevalence of age > 69 years old (12.46%) was greatly superior to that of 40–55 years old (4.26%) and 56–69 years old (6.24%) (*P* < 0.05), suggesting that the older the age is, the higher the risk of COPD. There were 61 patients with family history and 23 patients without a family history, and the prevalence rate of family history (44.53%) was greatly superior to that of no family history (2.73%), indicating that genetic susceptibility plays a very important role in the occurrence of COPD, which is conducive to explaining COPD at the genetic level. A multivariate logistic regression model was used to analyze the factors related to COPD. The regression coefficients of age, family history of COPD, and smoking were 0.557, 0.513, and 0.717, respectively (*P* < 0.05), suggesting that advanced age, family history of COPD, and smoking are independent risk factors for COPD.

To explore the early diagnostic value of CT images based on deep learning for COPD, an improved double residual convolutional neural network (DRCNN) model was employed to enhance CT images, and the CNN model and ResNet model were adopted for comparison. The results showed that the NMAD and PSNR of the DRCNN model were greatly superior to those of the CNN model and ResNet model, while the MSE of the DRCNN model was significantly lower than those of the CNN model and ResNet model, and the differences were considerable (*P* < 0.05), indicating that the improved DRCNN model proposed has a better effect on CT image noise reduction than the traditional model and has good application value [25, 26]. Then, the sensitivity, specificity, and accuracy of DRCN-based CT and single CT for COPD were calculated using the known results as the gold standard. The results showed that the diagnostic sensitivity, specificity, and accuracy of DRCN-based CT for COPD were greatly superior to those of single CT, and the difference was considerable (*P* < 0.05). This indicates that CT based on the DRCNN model can improve the diagnostic accuracy of simple CT images for COPD and has good performance in the early screening of COPD.

## 5. Conclusion

This research conducted a questionnaire survey on 980 permanent residents aged ≥ 40 years. Among them, 84 patients who were diagnosed with COPD and volunteered to participate in the experiment and 25 healthy people were selected as the research subjects, and all underwent CT imaging scans. At the same time, an image noise reduction model based on the DRCNN was proposed to process CT images. Finally, it was found that CT based on the DRCNN model can improve the diagnostic accuracy of COPD by simple CT images and has a better performance in the early screening of COPD. Old age, family history of COPD, and smoking were independent risk factors for COPD. However, the samples included in this study were all from one hospital, which had geographical limitations. Moreover, the risk factors for COPD have not been fully included, such as passive smoking, years of use of firewood, and exposure history of occupational dust, so more risk factors will be included in the subsequent study for discussion. In conclusion, this study provides a data reference for related factors and imaging examinations of COPD.

## Figures and Tables

**Figure 1:** Image processing flow of the DRCNN model.

**Figure 2:** General data of the investigation samples. (a)–(h) were sex, smoking, age, education level, marital status, BMI, family history of COPD, and heating method, respectively.

**Figure 3:** Comparison of prevalence rates under different sociological data. (a)–(h) gender, smoking, age, education level, marital status, BMI, family history of COPD, and heating method, respectively. ^*∗*^ indicates that there were statistically significant differences between men and women, between smokers and nonsmokers, between different ages, between people with different BMI, and between those with or without a family history (*P* < 0.05).

**Figure 4:** Comparison of performance indexes of different algorithms. (a)–(c) NMAD, MSE, and PSNR, respectively. ^*∗*^ compares with the DRCNN model, *P* < 0.05.

**Figure 5:** CT image processing effects of different algorithms. (a)–(d) the original image, CNN model processed image, ResNet model processed image, and DRCNN model processed image, respectively.

**Figure 6:** CT image data of a patient with COPD. Male, 75 years old, cough, shortness of breath, bloody expectoration, and sometimes unable to breathe and woke up at night.

**Figure 7:** Comparison of diagnostic results between DRCN-based CT and single CT (a)–(c) sensitivity, specificity, and accuracy, respectively; 1 is CT based on the DRCNN model; 2 is single CT. ^*∗*^ compared with 1, *P* < 0.05.

**Table 1:** Multivariate logistic regression analysis of COPD occurrence.

The independent variables	Regression coefficient	*t*	*P*
Gender	0.434	5.054	0.051
Age	0.557	4.592	0.000
BMI	0.262	4.027	0.078
Family history of COPD	0.513	5.822	0.000
Smoking	0.717	4.933	0.018

## Data Availability

The data used to support the findings of this study are available from the corresponding author upon request.
